# Early cognitive function, recovery and well-being after sevoflurane and xenon anaesthesia in the elderly: a double-blinded randomized controlled trial

**DOI:** 10.1186/2045-9912-1-9

**Published:** 2011-05-18

**Authors:** Jan Cremer, Christian Stoppe, Astrid V Fahlenkamp, Gereon Schälte, Steffen Rex, Rolf Rossaint, Mark Coburn

**Affiliations:** 1 Department of Anaesthesiology, University Hospital Aachen of the RWTH Aachen, Pauwelsstraße 30, D-52074 Aachen, Germany

## Abstract

**Background:**

The postoperative cognitive function is impaired in elderly patients after general anaesthesia. The fast recovery after xenon anaesthesia was hypothesized to be advantageous in this scenario. We compared early postoperative cognitive function after xenon and sevoflurane anaesthesia in this study.

**Methods:**

The study was approved by the local ethics committee and written informed consent was obtained from each patient. Patients aged 65-75 years (ASA I-III) scheduled for elective surgery (duration 60-180 min) were enrolled. Investigators performing cognitive testing and patients were blinded towards allocation to either xenon or sevoflurane anaesthesia. Baseline assessment of cognitive function was carried out 12-24 h before the operation. The results were compared to follow-up tests 6-12 and 66-72 h after surgery. Primary outcome parameter was the subtest "Alertness" of the computerized Test of Attentional Performance (TAP). Secondary outcome parameters included further subtests of the TAP, several Paper-Pencil-Tests, emergence times from anaesthesia, modified Aldrete scores and patients' well-being.

**Results:**

40 patients were randomized and equally allocated to both groups. No significant differences were found in the TAP or the Paper-Pencil-Tests at 6-12 and 66-72 h after the operation. All emergence times were faster after xenon anaesthesia. The modified Aldrete scores were significantly higher during the first hour in the xenon group. No difference in well-being could be detected between both groups.

**Conclusions:**

The results show no difference in the incidence of postoperative cognitive dysfunction (POCD) after xenon or sevoflurane anaesthesia. Emergence from general anaesthesia was faster in the xenon group.

## Introduction

Age is a known risk factor for postoperative cognitive dysfunction (POCD) after cardiac and non-cardiac surgery [1-3]. Up to 41% of patients aged 60 years and older are affected by POCD and exposed to an increased risk of death within the first 12 months after major non-cardiac surgery [1].

Although a growing number of researchers are concentrating on POCD [4], no significant progress can be seen in the prevention of POCD.

The noble gas xenon offers good haemodynamic stability [5-10] and favours rapid recovery from anaesthesia [11,12], both of which have been hypothesized to be beneficiary in the reduction of POCD [13-15]. Xenon is a safe anaesthetic agent [12,16,17] which has been approved for clinical use in Germany (ASA I-III patients) since 2005 and in Europe (ASA I-II patients) since 2007 [18]. Its remarkable potential of neuronal protection has been demonstrated in several *in vivo *and *in vitro *models of ischemic and traumatic neuronal injury [19-24].

This study was conducted to investigate early postoperative cognitive function in elderly patients after general anaesthesia, hypothesizing a positive influence by use of xenon compared to sevoflurane.

Confirmation of this hypothesis would be an important step towards establishing strategies for the prevention and reduction of POCD.

## Methods

The study was designed as a prospective, inpatient, double-blinded, randomized, controlled trial. It was conducted at the University Hospital Aachen, Germany after obtaining approval from the local ethics committee.

Random assignment of the patients to either the sevoflurane or xenon anaesthesia group was achieved by using a computer-generated allocation sequence. Study investigators and patients were blinded in terms of group assignment. It was not feasible to blind the anaesthetist due to the different administration methods of the anaesthetics.

Primary outcome parameter of this study was the cognitive function, which was assessed with the subtest "Alertness" of the computerized Test for Attentional Performance (TAP, Version 1.7; Psytest, 2002).

As described previously, several other subtests of the TAP and additional Paper-Pencil-Tests were selected to monitor a wide spectrum of cognitive functions [13,15,25,26].

The set of Paper-Pencil-Tests included the Digit-Symbol-Substitution-Test (DSST), Recall of Digit Span (DS) and the Trail Making Tests A and B [27-29].

Anxiety and Depression were measured with the Well-being Test Bf-S and the short form of the Spielberger State-Trait Anxiety Inventory (STAI) [30,31].

Secondary outcome parameters were the emergence times from anaesthesia and the modified Aldrete scores recorded in the post-anaesthetic care unit (PACU) [32]. Levels of vigilance, well-being and energy were also assessed in the PACU.

Patients were assessed for eligibility and gave informed written consent to participating in the trial. A total of 40 patients, aged 65-75 years, and ASA status I-III were enrolled in this study. Patients were excluded from the trial in case of diabetes mellitus, congestive heart failure, adrenal insufficiency, reduced renal and/or hepatic function, chronic alcohol or drug abuse, disabling neuropsychiatric disorders, increased intracranial pressure, a history of stroke, cardiopulmonary resuscitation or brain trauma within the past 12 months, anaphylactic reactions to anaesthetics, legal incapacity, a lack of cooperation or the need for emergency operations.

The elective surgical operations under general anaesthesia were planned for 60-180 min and scheduled in urology, gynaecology, neurosurgery, trauma, ENT, orthopaedics and abdominal surgery. Neurosurgery was limited to interventions on the spine.

Management of anaesthesia followed standardised instructions, identical for both groups. Following a 3 min period of preoxygenation (100% O_2_), anaesthesia was induced through a single slow i.v. injection of propofol (2 mg kg^-1^) and simultaneous infusion of remifentanil (0.5 μg kg^-1 ^over 60 s). Facilitation of tracheal intubation was achieved with rocuronium (0.6 mg kg^-1^).

Standard monitoring of the patients included pulse oximetry, three-lead ECG, non-invasive blood pressure, temperature (AS/3 monitor, GE Datex-Ohmeda, Helsinki, Finland), bispectral index monitoring (BIS Model A 2000^®^, Software Version 2.21, Aspect Medical Systems, Boston, MA, USA) and end-tidal concentrations of oxygen, carbon dioxide and anaesthetic gases. All parameters were recorded at fixed intervals of 5 min.

Maintenance of anaesthesia was achieved by either xenon or sevoflurane. Administration of sevoflurane was started with age-adapted equipotent MAC values of 1 with 1.1-1.4 vol% in 30% oxygen (Cato^®^, Draeger, Lübeck, Germany) [33].

Xenon was started at 60% xenon in 30% oxygen and administered with a close circuit anaesthesia machine (Physioflex^®^, Draeger, Lübeck, Germany) using a software modification to allow the reduction of xenon consumption under minimal flow conditions. The inspiratory concentration of xenon was measured with an automatically calibrated thermo-conductive device in the anaesthesia machine (± 3 vol% accuracy).

Air Liquide Deutschland GmbH (Business Unit, Krefeld, Germany) provided xenon of medical quality in steel cylinders for this study.

Infusion of remifentanil was carried out at a base rate of 0.15 μg kg^-1 ^min^-1 ^and titrated according to clinical needs. The remifentanil infusion was increased based on haemodynamic (heart rate, systolic arterial blood pressure), somatic (swallowing, movement) and autonomic sings (flushing, sweating, salivating) at 0.05 μg kg^-1 ^min^-1 ^increments until symptoms were resolved.

Standard treatment of blood loss and fluid replacement strategy were used if necessary.

The standardised instructions included the administration of piritramide 0.05 μg kg^-1 ^twenty minutes before the estimated end of surgery as well as a short infusion of metamizole 15 mg kg^-1^, both as part of the post-anaesthetic pain management.

Inhaled anaesthetics were reduced to 0.5 MAC ten minutes before the estimated end of the intervention.

Discontinuation of anaesthesia required completion of all surgical tasks (including bandaging) and complete recovery from neuromuscular block (TOF-Watch SX^®^, Organon Teknika, Eppelheim, Germany).

The return of spontaneous breathing was aided by allowing a rise of end-expiratory carbon dioxide levels up to 6.6 kPa.

Extubation of the patients' tracheas required full recovery of the upper airway reflexes, sufficient spontaneous breathing (>8 breaths min^-1^, SaO_2 _> 95% with F_i_O_2 _at 100%) and haemodynamic stability.

Starting with the discontinuation of the anaesthetic, a blinded investigator recorded the emergence times from anaesthesia as part of the secondary outcome parameters. This included the time to extubation, time to awakening (eyes open), time to basic verbal command (squeeze investigator's hand) and time to return of orientation (date, time, place), all determined at 20 s intervals.

All patients were transferred from the operating room to the post-anaesthetic care unit for recovery. The study investigator recorded the modified 10-point scaled Aldrete scores at 5, 15, 30, 45, 60 min and at discharge from the PACU.

Pain level, dosage of postoperative analgesics, incidence of nausea and vomiting, use and dosage of antiemetics, as well as vigilance, well-being and energy were rated and recorded at the same intervals. Pain management included piritramide 0.05 mg kg^-1 ^if VAS for pain was rated >3.

The primary outcome parameter, as well as the additional measures of cognitive function, was recorded for each patient during three predetermined time intervals. Baseline testing was completed 12-24 h preoperatively. These tests were repeated in the same order between 6-12 h and again after 66-72 h postoperatively.

All instructions on how to perform the tests were given in a standard way by a blinded investigator to ensure uniform collection of data. The assessment took place in a quiet room, reducing outside disturbances. The tests were completed by the patients in about 45-60 min.

The TAP consists of low complexity tasks, using easily distinguishable stimuli that demand a simple motor response from the patient. It is designed to reduce interfering factors, such as sensory and motor failure and disturbances of speech or memory. The test batteries consisted of the subtests for Alertness, Visual Scanning, Divided Attention, Reaction Change and Working Memory. All tests were administered at the highest level of difficulty.

The two groups were compared in terms of test performance normalized to the preoperative baseline assessment and in terms of the number of patients with a decrease of 20% or more in test performance. A patient with a 20% decrease in at least 20% of all tests was considered to be suffering from POCD [15,34].

During the 6-12 h postoperative assessment, patients were asked to evaluate the anaesthesia and questioned whether they would choose the same procedure for further operations.

Statistical analysis was performed using SPSS 16.0 (SPSS Inc., Chicago, IL, USA); all figures were generated with GraphPad PRISM^® ^(GraphPad Software Inc., La Jolla, CA, USA). Categorical data were tested with the two-tailed Fisher's exact test and are presented as numbers and per cents of total. Parametric data were analysed with one-way ANOVA and are given accordingly as means and standard error of the means, means and 95% confidence intervals, means and standard deviation or means and range.

The sample size of this study was calculated for the primary outcome parameter (subtest "Alertness" of the TAP) with a significance level of α = 0.05 and a power of β = 0.8, considering a difference of 20% as relevant. Mean values and standard deviations of the primary outcome parameter were taken from the TAP databases (patients ≥ 65 years; n = 416; 242 ± 60 ms). The trial size was calculated with n = 18 and then determined with n = 20 patients per group to compensate for possible dropouts. The power calculation was performed with nQuery Advisor^®^, Version 7.0 (Statistical Solutions, Saugus, MA, USA).

## Results

A total of 40 patients were included in this study, equally distributed between the two groups. 39 patients underwent baseline testing prior to the operation and 37 patients completed the 6-12 h postoperative assessment (18 from the sevoflurane and 19 from the xenon group), while the 66-72 h assessment was completed by 18 and 14 patients (32 in total). The reasons for drop-outs included refusal of testing and discharge from the hospital previous to assessment and are shown in Figure 1.

**Figure 1:** **Flowchart**. Flowchart showing patients during the course of the trial, including reasons for dropouts.

The study groups were comparable regarding the distribution of patients' age, weight and height, level of education, gender, Apfel-Score and ASA status (Table 1).

**Table 1:** Patient data

	Sevoflurane (n = 20)	Xenon (n = 19)	*P*-value
Age (years)	70 (65-75)	69 (65-75)	0,441
Height (cm)	169 (9)	171 (6)	0,461
Weight (kg)	78 (12)	78 (12)	0,906
Gender male/female	11/9	13/6	0,514
Education <12/≥12 yr	17/3	15/4	0,469
ASA I/II/III	1/13/6	0/13/6	0,614
Apfel-Score 1/2/3/4	8/8/3/1	9/8/2/0	0,745

Age is presented as mean (range). Height and weight of the patients are given as mean (SD). Gender, school education <12 or ≥12 years, ASA classification and Apfel-Score are presented in total numbers.

Baseline-testing was scheduled 12-24 h prior to the operation and all patients underwent testing within that time-frame. The mean time-point of baseline-testing was at 18:33 (18:12-18:54) in the sevoflurane group and at 17:54 (17:30-18:18) in the xenon group, resulting in a difference between the two groups (Table 2).

**Table 2:** Anaesthesia data and times of testing

	Sevoflurane	Xenon	*P*-value
Average gas concentration (%)	1,18 (0,2)	53 (5,2)	-
Type of surgery			
Trauma	3 (15)	2 (10,5)	0,967
Orthopaedics	2 (10)	2 (10,5)	
ENT	1 (5)	1 (5,3)	
Gynaecology	2 (10)	3 (15,8)	
Urology	7 (35)	7 (36,8)	
Neurosurgery	4 (20)	4 (21,1)	
Abdominal surgery	1 (5)	0 (0)	
Anaesthesia time (min)	151 (121-181)	164 (121-206)	0,606
PACU time (min)	65 (52-79)	78 (64-93)	0,186
Remifentanil consumption (μg/kg/min)	0,13 (0,05)	0,16 (0,04)	0,065
Intraoperative piritramide (mg)	5,9 (2,4)	5,6 (1,2)	0,364
Postoperative piritramide (mg)	7,9 (4,7)	5,8 (4,2)	0,625
Preoperative assessment (hh:min)	18:33 (18:12-18:54)	17:54 (17:30-18:18)	0,016
6-12 h postop. assessment (hh:min)	15:42 (13:42-17:42)	15:15 (13:10-17:21)	0,746
66-72 h postop. assessment (hh:min)	15:39 (13:51-17:27)	15:36 (14:12-17:00)	0,969

Average anaesthetic gas concentration is displayed as mean (SD). Type of surgery is presented in number (% of total). Anaesthesia and PACU times are given as means with the upper and lower 95% confidence interval in parentheses. Remifentanil values and intra- and postoperative consumption of piritramide are presented as means (SD). Time points of pre- and postoperative testing are shown in hours and minutes with the upper and lower 95% confidence interval in parentheses.

Duration of anaesthesia as well as the type of surgery did not differ between groups. The average end-tidal concentration of volatile anaesthetics for maintenance of anaesthesia was 1.18% (0.2) for sevoflurane and 53% (5.2) for xenon. Consumption of remifentanil (intraoperative) and piritramide (intra- and postoperative) were comparable between the two groups.

All recovery-times recorded during the emergence from anaesthesia showed a difference between groups regarding "time to open eyes", "time to react on demand", "time to extubation" and "time to time and spatial orientation" with a significantly faster recovery in the xenon group (Table 3).

**Table 3:** Emergence from anaesthesia

Time	Sevoflurane	Xenon	*P*-value
to open eyes	8,5 (6,7-10,3)	4,6 (3,8-5,5)	≤0,001
to react on demand	8,0 (6,1-9,9)	4,6 (3,5-5,7)	0,004
to extubation	8,3 (6,5-10,1)	4,6 (3,8-5,5)	0,001
to time and spatial orientation	10,3 (8,7-11,8)	7,6 (6,1-9,1)	0,014

All times are given in minutes as mean with lower and upper 95% confidence interval in parentheses.

There was no significant difference in the length of stay in the PACU (Table 2). The modified Aldrete scores recorded in the PACU were significantly higher in the xenon group from arrival until 60 min, while results at discharge were comparable. The following other scores from the PACU were in favour of xenon: vigilance at 5 min; well-being at 30 and 45 min and energy during the complete period (Table 4).

**Table 4:** PACU data

	Sevoflurane	Xenon	*P*-value
Aldrete A	8,9 (0,9)	9,7 (0,6)	0,007
Aldrete 5	8,9 (1,0)	9,7 (0,5)	0,005
Aldrete 15	9,1 (1,0)	9,7 (0,6)	0,023
Aldrete 30	9,2 (1,1)	9,8 (0,3)	0,028
Aldrete 45	9,1 (1,1)	9,9 (0,3)	0,01
Aldrete 60	9,1 (1,1)	9,9 (0,4)	0,034
Aldrete D	9,8 (0,4)	9,7 (0,7)	0,88
Vigilance A (A/T/S)	7/12/1 (35/60/5)	13/5/0 (72/287/0)	0,061
Vigilance 5 (A/T/S)	9/11/0 (45/55/0)	15/3/0 (83/17/0)	0,014
Vigilance 15 (A/T/S)	10/10/0 (50/50/0)	13/5/0 (72/28/0)	0,162
Vigilance 30 (A/T/S)	12/8/0 (60/40/0)	14/4/0 (78/22/0)	0,239
Vigilance 45 (A/T/S)	9/7/0 (56/44/0)	13/4/0 (76/24/0)	0,218
Vigilance 60 (A/T/S)	6/5/0 (55/45/0)	10/3/0 (77/23/0)	0,247
Vigilance D (A/T/S)	16/4/0 (80/20/0)	17/1/0 (94/6/0)	0,188
Well-being A (E/G/F/P)	0/5/10/5 (0/25/50/25)	0/10/5/2 (0/59/29/12)	0,111
Well-being 5 (E/G/F/P)	0/5/10/5 (0/25/50/25)	1/9/5/2 (6/53/29/12)	0,18
Well-being 15 (E/G/F/P)	0/6/10/4 (0/30/50/20)	0/11/5/1 (0/65/29/6)	0,094
Well-being 30 (E/G/F/P)	0/5/11/4 (0/25/55/20)	0/11/6/0 (0/65/35/0	0,023
Well-being 45 (E/G/F/P)	0/3/10/3 (0/19/62/19)	0/10/6/0 (0/62/38/0)	0,021
Well-being 60 (E/G/F/P)	0/3/8/0 (0/27/73/0)	0/6/6/0 (0/50/50/0)	0,265
Well-being D (E/G/F/P)	0/7/13/0 (0/35/65/0)	0/11/7/0 (0/61/39/0)	0,07
Energy A (N/F/P)	0/5/15 (0/25/75)	3/11/4 (17/61/22)	0,003
Energy 5 (N/F/P)	0/5/15 (0/25/75)	2/12/4 (11/67/22)	0,004
Energy 15 (N/F/P)	0/8/12 (0/40/60)	2/13/3 (11/72/17)	0,014
Energy 30 (N/F/P)	1/8/11 (5/40/55)	2/15/1 (11/83/6)	0,005
Energy 45 (N/F/P)	0/6/10 (0/38/62)	3/14/0 (18/82/0)	≤0,001
Energy 60 (N/F/P)	0/5/6 (0/45/55)	2/11/0 (15/85/0)	0,006
Energy D (N/F/P)	2/9/9 (10/45/45)	3/15/0 (17/83/0)	0,005

All values were recorded at the PACU upon arrival (A), after 5 (5), 15 (15), 30 (30), 45 (45), 60 (60) minutes and at discharge (D). Modified Aldrete scores are given as mean (SD). Vigilance, Well-being and Energy are shown in total numbers (% of total). Vigilance was distinguished as awake (A), tired (T) or sleeping (S). Well-being was rated as excellent (E), good (G), fair (F) or poor (P). Energy was classified as normal (N), fair (F) or poor (P).

Both postoperative assessments were performed at similar time points (Table 2). The results of patients' self-evaluation of the anaesthesia were homogenous in both groups.

There were no differences between the two groups at the 12-24 h preoperative baseline assessment of cognitive function with the TAP and the Paper-Pencil-Tests. The postoperative tests at 6-8 and 66-72 h were normalized to the preoperative baselines.

The subtest "Alertness" as the primary outcome parameter of this study, as well as all other subtests of the TAP and the Paper-Pencil-Tests, did not show a significant difference between the two groups (Figures 2 + 3).

**Figure 2:** **TAP**. Cognitive function assessed with the TAP. Subtests Alertness (A+B), Divided Attention (C+D), Visual Scanning (E+F), Working Memory (G+H) and Reaction Change (I+J). Figure pairs show reaction time on the left and valid reactions on the right. All values are Mean (SEM) and display the change at 6-8 and 66-72 hours normalized to the preoperative baseline. All ordinates are in per cent. Grey lines and open circles display the xenon group, black lines and open squares represent the sevoflurane group.

**Figure 3:** **Well-being and Paper-Pencil-Tests**. Well-being measured with Bf-S (A) and STAI (B), cognitive function assessed with Paper-Pencil-Tests DS (C), DSST (D), Trail Making Test A and B (E+F). An increase in percent shows a decline in well-being (A+B) and a decline in outcome for E and F. A decrease in percent in C and D shows an increase in outcome. All values are Mean (SEM) and display the change at 6-8 and 66-72 hours normalized to the preoperative baseline. All ordinates are in percent. Grey lines and open circles display the xenon group, black lines and open squares represent the sevoflurane group.

The number of patients with a decline of 20% or more in test performance is shown for each test in Table 5. The Trail Making Test A conducted at 66-72 h was the only test with a significant difference, while all other Paper-Pencil-Tests and the TAP showed no difference between the groups (Table 5).

**Table 5:** POCD

	6-8 h postoperative >20%			66-72 h postoperative >20%		
	
	Sevoflurane	Xenon	*P*-value	Sevoflurane	Xenon	*P*-value
DS	5 (26)	2 (11)	0,405	5 (28)	3 (21)	1
DSST	4 (21)	3 (17)	1	1 (6)	0 (0)	1
TMT A	4 (21)	4 (22)	1	1 (6)	6 (43)	0,027
TMT B	4 (21)	6 (33)	0,476	3 (17)	0 (0)	0,238
Alertness RT	5 (26)	4 (22)	1	2 (12)	2 (14)	1
Alertness VR	0 (0)	2 (11)	0,23	1 (6)	1 (7)	1
Divided Attention RT	2 (11)	1 (6)	1	1 (6)	2 (14)	0,576
Divided Attention VR	1 (6)	1 (6)	1	2 (12)	0 (0)	0,488
Visual Scanning RT	7 (37)	3 (17)	0,269	4 (25)	2 (14)	0,657
Visual Scanning VR	3 16)	3 (17)	1	3 (19)	2 (14)	1
Working Memory RT	3 (16)	4 (22)	0,693	5 (31)	3 (21)	0,689
Working Memory VR	5 (26)	5 (28)	1	1 (6)	0 (0)	1
Reaction Change RT	3 (16)	1 (6)	0,608	0 (0)	0 (0)	-
Reaction Change VR	0 (0)	2 (13)	0,202	0 (0)	1 (8)	0,433

Cognitive function assessed with Paper-Pencil-Tests and the TAP. Decline >20% to the 12-24 h preoperative values is presented in numbers (% of total). Paper-Pencil-Tests are Recall of Digit Span (DS), Digit-Symbol-Substitution-Test (DSST), Trail Making Test A and B (TMT A, TMT B). Subtests of the TAP were analyzed in terms of mean reaction time (RT) and number of valid reactions (VR).

Postoperative cognitive dysfunction was defined as a 20% decline in 20% of all tests (TAP and Paper-Pencil-Tests combined) [15,34]. The incidence was comparable between the two groups at the postoperative evaluations at 6-8 h (xenon 39%, sevoflurane 32%; *p *= 0.737) and 66-72 h (xenon 29%, sevoflurane 44%; *p *= 0.471).

A decrease in patients' well-being was measured with the Bf-S in both groups 6-12 h after the operation, while closely returning to baseline values at the second postoperative evaluation (Figure 3). Anxiety assessed with the STAI showed a continuous decrease during both postoperative assessments in all patients (Figure 3).

## Discussion

We compared early cognitive function in elderly patients after xenon or sevoflurane anaesthesia in this study.

None of the applied tests detected a significant difference in the incidence of POCD between the xenon and the sevoflurane group.

Selection of the correct testing instruments is essential, since the definition of POCD and its measurement varies in previous studies [4,35]. The TAP is a commonly used device to measure attention (further information: http://www.psytest.net) [13,15]. In this study, we used its subtests Alertness, Divided Attention, Visual Scanning, Working Memory and Reaction Change, along with several Paper-Pencil-Tests.

Repeated postoperative assessments might result in a learning effect. The retest reliability of the TAP was shown before [25], although our test intervals were much shorter in this study. The intervals were identical with those suggested by previous studies [13,15]. Alternating equivalent versions of the Paper-Pencil-Tests were used if available, in an effort to minimize learning effects [4,35].

The subtest "Alertness" of the TAP as the primary outcome parameter did not show a significant difference in test performance between the two groups. Additional subtests of the TAP enabled us to monitor a wider spectrum of cognitive functions, but also showed comparable results. The applied Paper-Pencil-Tests detected no difference in test performance.

The number of patients with a decrease of 20% or more was comparable for each test between the two groups, with exemption of the Trail Making Test A conducted at 66-72 h postoperatively. The relevance of this finding is limited due to the fact that this test is only one of twelve aspects considered in our calculation of actual postoperative cognitive dysfunction.

The over-all incidence of POCD was high, but comparable between the two groups at both postoperative evaluations (6-8 h: xenon 39%, sevoflurane 32%; 66-72 h: xenon 29%, sevoflurane 44%). Other studies found similar figures, but direct comparison with our study is limited due to the use of different tests and investigated substances [15,26,36].

We were able to show significant differences within each group in comparison to the preoperative baseline in some tests, but could not detect such differences between the two groups.

These findings are in accordance with previous studies [4,13,15,26]. None of the investigated anaesthesia regimens showed a significant benefit in terms of reduced incidence and severity of POCD. However all of these studies are limited in their power.

Preoperative testing is crucial, since all calculations are based on these results. The pending operation can pose a stress factor for the patients and hence possibly influence the test results. We chose a 12-24 h period prior to the operation for our assessment in an attempt to limit these effects in comparison to an assessment directly before premedication was given as used by Heavner and colleagues [14]. An earlier time-point would be preferable, but could not be realized in the clinical routine.

Considering the time-frame of 12 h for the assessment (12-24 h preoperatively), we felt that the difference of 39 min between the mean time-points of testing in the two groups would not have a relevant effect on the results. Variations in time-points of testing are the consequence of choosing a preoperative time-frame over a fixed time-point for the assessment. The actual impact can not be quantified, but we suspected a justifiable benefit from earlier testing.

The power was calculated for the primary outcome parameter, considering 20% as a relevant difference. As discussed in previous studies, 10-15% could be a clinically more relevant value [15]. Regarding the secondary outcome parameters and this consideration, the study might be underpowered.

The high drop-out rate in the xenon group before the second postoperative assessment could have further altered our results.

Sevoflurane was used with an average end-tidal concentration of 1.18% (0.2), which is equivalent to 75% of an age-adapted MAC according to Nickalls and Mapleson [33]. Xenon was used with a mean concentration of 53% (5.2), resembling 84.1% of a MAC. Since there are no age-adapted MAC values for xenon available, we presumed that the used gas concentrations were equivalent. They match the concentrations used in other studies [37,38].

The times recorded during recovery of anaesthesia were significantly faster in the xenon group. This corresponds with the low blood-gas partition coefficient of xenon (0.115) compared to sevoflurane (0.69) [11]. The results are similar to those described in earlier studies [13,15,17,39].

The scores from the PACU were partially in favour of xenon. The modified Aldrete-scores and the level of energy were higher in the xenon group throughout the recorded time-period. These results are comparable with previous findings [13,15].

The Aldrete-scores were homogenous in both groups at discharge from the PACU. Self-evaluation of the anaesthesia showed no difference between patients from the two groups. Patients' well-being showed a comparable development during the course of the trial (Figure 3).

## Conclusions

In conclusion, xenon anaesthesia enables significantly faster emergence from anaesthesia in the elderly.

No difference in the incidence of POCD could be detected after xenon and sevoflurane anaesthesia. The occurrence was comparable in both groups 6-8 and 66-72 h after the operation.

## Competing interests

This study was supported by Air Liquide Deutschland GmbH (donor of xenon).

MC and RR received lecture and consultant fees from Air Liquide Santé International, a company interested in developing clinical applications for medical gases, including xenon.

## Authors' contributions

JC and MC performed the statistical analysis and drafted the manuscript. MC and RR participated in the study design and coordination. AVF, CS, GS, JC and SR helped to perform the anaesthesia and revised the manuscript. All authors read and approved the final manuscript.
